# Thymic lymphoid hyperplasia with multilocular thymic cysts diagnosed before the Sjögren syndrome diagnosis

**DOI:** 10.1186/s13000-015-0332-y

**Published:** 2015-07-16

**Authors:** Hiroshi Minato, Eriko Kinoshita, Satoko Nakada, Takayuki Nojima, Makoto Tanaka, Katsuo Usuda, Motoyasu Sagawa, Haruka Iwao, Masao Tanaka, Mariko Doai, Tomoko Takahashi, Naoko Shibata

**Affiliations:** Department of Pathology and Laboratory Medicine, Kanazawa Medical University, 1-1 Daigaku, Uchinada, Kahoku, Ishikawa 9200293 Japan; Department of Thoracic Surgery, Kanazawa Medical University, Uchinada, Ishikawa Japan; Department of Hematology and Immunology, Kanazawa Medical University, Uchinada, Ishikawa Japan; Department of Radiology, Kanazawa Medical University, Uchinada, Ishikawa Japan; Department of Ophthalmology, Kanazawa Medical University, Uchinada, Ishikawa Japan

**Keywords:** Thymus, Multilocular thymic cysts, Lymphoid hyperplasia, Follicular hyperplasia, Sjögren syndrome, Immunohistochemistry

## Abstract

**Background:**

Thymic lymphoid hyperplasia is often present with myasthenia gravis as well as other autoimmune diseases such as systemic lupus erythematosus and rheumatoid arthritis. Of the 4 cases of thymic lymphoid hyperplasia associated with Sjögren syndrome that have been reported, no case with a thymic lesion diagnosis that led to the diagnosis of Sjögren syndrome has been reported. We herein report a case of thymic lymphoid hyperplasia with multilocular thymic cysts, diagnosed before Sjögren syndrome.

**Case presentation:**

A 37-year-old Japanese woman had an approximate 5-cm anterior mediastinal mass detected by chest imaging. The resected lesion revealed multilocular thymic cysts that were filled with colloid-like material. Histology showed lymph follicular hyperplasia with many epithelial cysts. The epithelium consisted of thymic medullary epithelium, and no epithelial proliferation was seen in the lymphoid tissue. Lymphocytes were composed of an organized mixed population of mature T and B cells without significant atypia. The infiltrated B cells did not reveal light chain restriction or immunoglobulin heavy chain gene rearrangement. After the pathological diagnosis of thymic lesion, tests for the presence of autoantibodies were positive for antinuclear antibodies, rheumatic factor, and anti-SSA/Ro antibodies. The Schirmer’s, chewing gum, and Saxon tests showed decreased salivary and lacrimal secretion. Lip biopsy showed focal lymphocytic sialadenitis. The signs and symptoms of Sjögren syndrome had not resolved, without aggravation, 1 year after the thymectomy.

**Conclusion:**

When a case with thymic lymphoid hyperplasia without myasthenia gravis is encountered, it is essential to consider the presence of another autoimmune disease including Sjögren syndrome.

## Background

Thymic lesions in Sjögren syndrome primarily consist of extranodal marginal zone B-cell (MALT) lymphoma and rarely consist of thymoma, thymic carcinoma, or lymphoid hyperplasia [1]. Of the 4 cases with thymic lymphoid hyperplasia associated with Sjögren syndrome that have been reported [1–3], 3 cases were accompanied by multilocular thymic cysts. We herein report a case of thymic lymphoid hyperplasia with multilocular thymic cysts that led to the diagnosis of preclinical Sjögren syndrome. To the best of our knowledge, a diagnosis of thymic lymphoid hyperplasia before the diagnosis of Sjögren syndrome has not previously been reported.

## Case presentation

A 37-year-old Japanese woman was referred to our hospital for general malaise. Chest radiography, computed tomography (CT), and magnetic resonance imaging revealed a superior anterior mediastinal tumor that was 4.7 × 3.8 × 2.8 cm in size, with multilocular cysts. CT with contrast enhancement showed mild enhancement of the septum of the lesion (Fig. 1a-c). T1-weighted and T2-weighted images revealed isointensity and high intensity, respectively, of the lesion (Fig. 1d). Calcification or fatty components were not seen. The positron emission tomography standardized uptake value (PET SUVmax) was 4.25, which was relatively low (Fig. 1e). The following tumor markers were all within normal range: carcinoembryonic antigen, alpha-fetoprotein, squamous cell carcinoma antigen, CYFRA 21–1, sialyl Lewis X, and progastrin-releasing peptide. Anti-acetylcholine receptor antibodies were not detected. Thymoma, thymic cyst, or teratoma was suspected, and a thymectomy was performed. After the pathological diagnosis, on suspicion of an associated autoimmune disease, autoantibodies were examined and were positive for antinuclear antibodies (speckled type, ×640), rheumatic factor (114; normal range <15 IU/mL), and anti-SSA/Ro antibodies (>240; normal <10 U/mL) and negative for anti-SS-B/La, anti-DNA, anti-RNP, anti-Sm, anti-cyclic citrullinated peptide, Jo-1, Scl-70, and anti-neutrophil cytoplasmic antibodies (MPO-ANCA and PR3-ANCA). She also had a mildly dry mouth and dry eyes. The Schirmer’s (right 2 mm/left 2 mm), chewing gum (2.9 mL/10 min), and Saxon (0.62 g/2 min) tests all showed decreased secretion of the lacrimal and salivary glands. A lip biopsy specimen revealed focal lymphocytic sialadenitis. Based on these findings, Sjögren syndrome was diagnosed. The signs and symptoms of Sjögren syndrome, without aggravation, were not resolved 1 year after the thymectomy, and autoantibody titers did not show remarkable changes.

**Fig. 1:** Radiological imaging of the lesion. Contrast-enhancement computed tomography (CT) shows a tumor in the superior anterior mediastinum with slightly enhanced multiple septa (**a**-**c**). Magnetic resonance imaging (MRI) with fat suppression reveals the tumor with high-intensity (**d**). The standardized uptake value (SUVmax) of positron emission tomography (PET)-CT was 4.25, which was relatively low (**e**)

### Pathological findings

The resected thymectomy specimen was 9.5 × 5.5 × 2.5 cm in size and weighed 61 g. An ill-defined elastic firm mass, 5 × 3.5 × 2.5 cm in size, was found in the thymus with multilocular cysts, many of which were filled with yellowish-green colloid-like material (Fig. 2). Histology of the tumor revealed lymphoid tissue with hyperplastic germinal centers and occasional Hassall corpuscles (Fig. 3). The cysts were lined by thin layers of thymic epithelium (Fig. 4). Outside the tumor in the thymus, there were many small nodules of lymphoid tissue showing similar morphology as the main tumorous lesion. In the small nodules of lymphoid tissue, microscopic cysts lined by thymic epithelium were occasionally found (Fig. 5). The lymphocytes were small and mature except for cells in germinal centers. No significant atypia was seen in the lymphoid and epithelial cells. Immunohistochemically, cytokeratin AE1/AE3 highlighted the epithelium of the cysts and Hassall corpuscles (Fig. 6). There was no epithelial proliferation in the nodular lymphoid tissue; the findings eliminated the possibility of thymoma. Lymphoid markers revealed organized mixed distribution of CD3+, CD5+, CD20+, and CD79+ cells and did not show monoclonal proliferation of B cells or T cells (Fig. 7a,b). Immunostaining of light chains showed that the approximate ratio of kappa to lambda was 3:1, and no significant light chain restriction was seen (Fig. 7c,d). Staining of immunoglobulin (Ig)G, IgA, and IgM heavy chains did not reveal monoclonal proliferation. Both CD20 + B cells and CD3 + T cells infiltrated the epithelium. No aberrant expression of CD5 and CD43 B cells was observed. Bcl-2 was negative in the germinal center of lymphoid follicles. Polymerase chain reaction and gene analysis from the formalin-fixed paraffin embedded tissue of the lesion did not show rearrangement of the immunoglobulin heavy chain (IgH) gene. Thymic lymphoid hyperplasia with multilocular thymic cysts was the pathological diagnosis.

**Fig. 2:** Macroscopic findings of the thymic tumor. An ill-defined tumor (5 × 3.5 × 2.5 cm) is seen in the upper part of the resected thymus (*arrow*) (**a**). The cut surface shows a multicystic tumor filled with yellowish-green colloid-like material (**b**)

**Fig. 3:** Histological findings of the thymic tumor. Lower power view shows the cystic walls are composed mostly of lymphoid tissue with epithelial linings. Cysts are filled with eosinophilic proteinous secretion containing cholesterol clefts

**Fig. 4:** Histologic findings of the cyst wall. Higher power view reveals that the cyst wall consists of mature small lymphocytes with a germinal center (*right lower*) and thymic medullary epithelium with Hassall corpuscles

**Fig. 5:** Histological findings of the thymus. Non-tumorous thymic tissue also shows hyperplastic lymphoid tissue with many germinal centers. Occasionally, microscopic cystic lesions (*right upper*) similar to the tumorous lesion are seen in the thymus

**Fig. 6:** Immunohistochemical findings of the epithelial marker. Immunohistochemistry of cytokeratin AE1/AE3 highlights the organized network of the thymic medullary epithelium surrounding hyperplastic lymphoid tissue. No epithelial proliferation is seen in the nodular lymphoid tissue

**Fig. 7:** Immunohistochemical findings of the lymphoid markers. Immunohistochemistry of CD3 (**a**) and CD20 (**b**) shows mixed distribution of T and B cells and does not show any monoclonal proliferation. Both CD20 + B cells and CD3+ T cells infiltrate the lining epithelium of the cyst. Immunostaining of light chains (**c**, **d**) does not show restriction of kappa (**c**) or lambda (**d**) chains

The lip biopsy specimen revealed mild atrophy of the minor salivary glands with mild fibrosis and focal lymphoid aggregation (Fig. 8). A lymphoepithelial lesion was not seen. The focus score [4] was 1.25 and was graded [5] as 4.

**Fig. 8:** Histological findings of the minor salivary gland. Histology of the labial minor salivary gland shows focal lymphocytic aggregation in the gland with mild glandular atrophy. A lymphoepithelial lesion is not seen. The focus score was 1.25 and was graded as 4

## Discussion

To the best of our knowledge, this is the first report of thymic lymphoid hyperplasia that led to the diagnosis of preclinical Sjögren syndrome. The lesion was accompanied by multilocular thymic cysts.

Thymic cysts are categorized as either congenital and acquired; the former is usually unicystic and non-inflammatory, and the latter is generally multicystic and associated with other diseases such as thymoma, thymic carcinoma, malignant lymphoma including MALT lymphoma, Hodgkin lymphoma, germ cell tumor, HIV infection, or lymphoid hyperplasia [1, 6]. Both unicystic and multicystic lesions are lined with flattened, cuboidal, ciliated columnar or stratified squamous epithelium, but multilocular thymic cysts are most likely the result of cystic transformation of medullary epithelium induced by an acquired inflammatory process [6]. The microscopic cysts found in the non-tumorous area of the present case suggest the beginning of such an acquired process.

Although the occurrence of thymic lymphoid hyperplasia is relatively rare, it is most commonly associated with myasthenia gravis (MG). Aside from MG, thymic lymphoid hyperplasia is most often accompanied with other autoimmune diseases such as systemic lupus erythematosus, rheumatoid arthritis, scleroderma, Sjögren syndrome, allergic vasculitis, and Hashimoto thyroiditis [1, 7]. In contrast to true thymic hyperplasia, thymic lymphoid hyperplasia usually does not show thymic enlargement but an increased number of lymphoid follicles [7]. Numerous hyperplastic germinal centers with tingible body macrophages and centroblastic and centrocytic cells are usually present [8]. The mantle zone is well defined, while the marginal zone is not developed. A normal thymic cortex is observed around the areas of lymphoid hyperplasia, and effacement of the thymic architecture with cortical atrophy is not seen. Differentiation from MALT lymphoma, Castleman disease, and lymphocyte predominant thymoma (type B1) is important.

In MALT lymphoma, interfollicular expansion of centrocyte-like cells, monocytoid B-cells, or plasmacytoid cells fill the medullary spaces and partially infiltrate reactive follicles (follicular colonization) with atrophic mantle zones. Nuclei of infiltrating lymphocytes are irregular with dense chromatin and occasional blastoid larger cells. These findings were not observed in the present case. Furthermore, each follicle is not surrounded by an epithelial network, as observed in the present case, and invasion of monocytoid B-cells or centrocyte-like lymphocytes with irregular nuclei are observed in MALT lymphoma. The present case did not have monoclonal proliferation of lymphocytes and plasma cells, and the genetic analysis from the formalin-fixed paraffin embedded tissue of the lesion did not show rearrangement of the IgH gene.

A hyaline vascular type of Castleman disease typically shows germinal centers containing a few small vessels bridging through to perifollicular tissue and is surrounded by concentrically arranged small lymphoid cells, whereas a plasma cell type shows diffuse sheet-like infiltration of plasma cells in the interfollicular zone. The present case did not show the typical histopathological changes of either type of Castleman disease.

A literature search in the PubMed database resulted in 22 cases of MALT lymphoma, 6 cases of thymoma, 4 cases of lymphoid hyperplasia, and 1 case of thymic carcinoma associated with Sjögren syndrome. Of the 4 cases of thymic lymphoid hyperplasia associated with Sjögren syndrome [1–3], 3 cases were accompanied by multilocular thymic cysts [1, 3]. To the best of our knowledge, a diagnosis of thymic lymphoid hyperplasia before the Sjögren syndrome diagnosis has not been reported previously. Although the preoperative signs and symptoms were mild, the patient fulfilled the criteria of primary Sjögren syndrome [9], including decreased secretion of the lacrimal and salivary glands, presence of autoantibodies to SSA/Ro, and a focus score >1 for the lip biopsy [10]. The patient had no history of other collagen vascular diseases, radiation therapy, hepatitis C infection, acquired immunodeficiency disease, malignant lymphoma, sarcoidosis, graft-versus-host disease, or use of anticholinergic drugs.

Although thymectomy leads to remission in a significant number of MG patients with thymic lymphoid hyperplasia [11–13], the disease outcome differs [11–13], especially in those with different types of autoantibodies [11]. Thymectomy did not appear to improve the sicca symptoms or to decrease the serum level of anti-SSA/Ro antigens in the present patient. Izumi, et al. [1] reported that the serum ANA levels remained high after thymectomy in two patients with Sjögren syndrome and thymic follicular hyperplasia, although without aggravation of their condition. We do not know which came first, the thymic lesion or Sjögren syndrome. Based on the experience of these few cases, Sjögren syndrome might develop first. However, even if the thymic lesion develops first, resection of thymic lesions might not improve, or only gradually improve, the autoimmune diseases that show poor response to corticosteroids, when compared with MG [14].

## Conclusions

We report a case of thymic lymphoid hyperplasia with multilocular thymic cysts, which led to the diagnosis of preclinical Sjögren syndrome. When we encounter a case with thymic lymphoid hyperplasia, we should consider the presence of autoimmune diseases. The precise mechanism underlying the association between Sjögren syndrome and thymic lesions is yet to be determined.

## Consent

Written informed consent was obtained from the patient for publication of this Case Report and any accompanying images. A copy of the written consent is available for review by the Editor-in-Chief of this journal.

## Abbreviations

MALT lymphoma: Extranodal marginal zone B-cell lymphoma
CT: Computed tomography
PET SUVmax: Positron emission tomography standardized uptake values
Ig: Immunoglobulin
IgH: Immunoglobulin heavy chain
MG: Myasthenia gravis
